The article "Cecal Lipoma: A Rare Etiology of Acute Appendicitis in Adults" was retracted in 2024. Reasons: content taken from a thesis; false authorship; unreliable results or conclusions; no approval from an author.

# Cecal Lipoma: A Rare Etiology of Acute Appendicitis in Adults

**DOI:** 10.7759/cureus.19423

**Published:** 2021-11-09

**Authors:** Yahya A Alnashri, Aali M Alhuzali, Eyyad A Edrees, Razan A Almuraykhi, Reem A Majrashi, Raghad A Alhomidan, Sarah B Alharbi, Farah A Alassaf, Aishah N Alsuhaibani, Rami S Sufyani, Ahmed S Alkhars, Maisa M Mallawi, Rawan Y Alkhotani, Mustafa M Qattan, Malak Alshammari

**Affiliations:** 1 College of Medicine, Umm Al-Qura University, Mecca, SAU; 2 College of Medicine, Imam Mohammad Ibn Saud Islamic University, Riyadh, SAU; 3 College of Medicine, Najran University, Najran, SAU; 4 College of Medicine, Qassim University, Qassim, SAU; 5 Medicine, King Salman Abdul Aziz Medical City, Madinah, SAU; 6 College of Medicine, Imam Abdulrahman Bin Faisal University, Dammam, SAU; 7 College of Medicine, Ibn Sina National College For Medical Studies, Jeddah, SAU

**Keywords:** case report, laparoscopy, lipoma, acute appendicitis, acute abdominal pain

## Abstract

Acute appendicitis is the most common indication for abdominal surgeries worldwide. Obstruction of the appendiceal orifice is thought to be the primary pathology of appendicitis. The obstruction leads to an increase in the intraluminal pressure resulting in ischemia and inflammatory process. Several pathologies could cause obstruction of the appendix lumen. These pathologies include hard fecal masses, stones, lymphoid hyperplasia, and neoplasia. We present the case of a 42-year-old man who presented to the emergency department with a complaint of abdominal pain and diarrhea for 3 days. The abdominal pain started in the periumbilical region and was shifted to the right lower quadrant of the abdomen. The pain started gradually and had been progressing in severity. He described the pain as a stabbing in nature. Abdominal examination revealed a soft abdomen with diffuse tenderness. However, the tenderness was more pronounced in the right iliac fossa with a positive rebound sign. Further, the Rovsing sign was positive. Initial laboratory investigation revealed elevated leukocyte count and elevated inflammatory markers, including erythrocyte sedimentation rate and C-reactive protein. The CT scan demonstrated well-defined homogenous fat density endoluminal lesion in the cecum with an average size of 6 cm with associated thickened wall appendix. The patient was prepared for an emergency laparoscopy for limited segmental rection of the cecum with appendectomy. Lipoma is a rare benign tumor of the gastrointestinal tract. Clinicians should maintain a high index of suspicion for benign and malignant neoplasms when they encounter patients with suspected acute appendicitis in the adult population.

## Introduction

Acute appendicitis is the most common indication for abdominal surgeries worldwide. Acute appendicitis is more frequent in the second and third decades of life, it can develop at any age [1]. Obstruction of the appendiceal orifice is thought to be the primary pathology of appendicitis. The obstruction leads to an increase in the intraluminal pressure resulting in ischemia and inflammatory process. However, the obstruction is not identified in all cases of acute appendicitis. For example, Arnbjörnsson and Bengmark revealed that only one-third of patients with acute appendicitis had elevated intraluminal pressure suggestive of obstruction [2]. Several pathologies could obstruct the appendix lumen. These pathologies include hard fecal masses, stones, lymphoid hyperplasia, and neoplasia. The pathologies causing acute appendicitis are strongly related to the age of the patient [1]. For instance, children tend to develop acute appendicitis due to lymphoid follicular hyperplasia while elderly patients may develop acute appendicitis because of obstructive malignancies. A variety of infectious and inflammatory conditions could give clinical pictures similar to that of acute appendicitis. Hence, imaging plays a crucial role in confirming the diagnosis [3]. Here, we present the case of a middle-aged man with right iliac fossa pain suggestive of acute appendicitis. The patient underwent a CT scan to confirm the diagnosis and has demonstrated a partially obstructive cecal lipoma associated with acute appendicitis.

## Case presentation

We present the case of a 42-year-old man who presented to the emergency department with a complaint of abdominal pain and diarrhea for 3 days. The abdominal pain started in the periumbilical region and was shifted to the right lower quadrant of the abdomen. The pain started gradually and had been progressing in severity. He described the pain as a stabbing in nature. It was exacerbated by movement and food intake. The pain was partially relieved by oral analgesic medications like paracetamol. The pain was associated with low-grade fever and decreased appetite. The patient also complained of diarrhea with five bowel motions/day. The stools were watery with no mucus or blood. He reported that diarrhea developed after he received an oral antibiotic therapy (cefuroxime) for a recent upper respiratory tract infection.

The past medical history of the patient was remarkable for diabetes mellitus that was well-controlled with oral antidiabetic agents. He did not undergo any previous abdominal surgeries. He had a smoking history of 15 pack-years. He had never drunk alcohol before. He worked as a taxi driver. The family history was unremarkable for any inherited gastrointestinal disorders.

Upon examination, the patient appeared sick. He was not pale, jaundiced, or cyanosed. Vital signs revealed tachycardia (115 bpm), low-grade fever (37.5℃), normal respiratory rate (14 bpm), and maintained blood pressure (122/80 mmHg). The oxygen saturation was 99% on room air. Abdominal examination revealed a soft abdomen with diffuse tenderness. However, the tenderness was more pronounced in the right iliac fossa with a positive rebound sign. Further, the Rovsing sign was positive. Initial laboratory investigation revealed elevated leukocyte count and elevated inflammatory markers, including erythrocyte sedimentation rate and C-reactive protein. The renal and hepatic profiles were within the normal limits (Table 1).

**Table 1:** Summary of the results of laboratory findings

Laboratory Investigation	Unit	Result	Reference Range
Hemoglobin	g/dL	14.5	13.0–18.0
White blood cell	1000/mL	14.2	4.0–11.0
Platelet	1000/mL	380	140–450
Erythrocyte sedimentation rate	mm/hr	25	0–20
C-reactive protein	mg/dL	14.0	0.3–10.0
Total bilirubin	mg/dL	0.8	0.2–1.2
Albumin	g/dL	3.9	3.4–5.0
Alkaline phosphatase	U/L	44	46–116
Gamma-glutamyltransferase	U/L	75	15–85
Alanine transferase	U/L	55	14–63
Aspartate transferase	U/L	28	15–37
Blood urea nitrogen	mg/dL	15	7–18
Creatinine	mg/dL	1.0	0.7–1.3
Sodium	mEq/L	138	136–145
Potassium	mEq/L	3.8	3.5–5.1
Chloride	mEq/L	104	98–107

In light of the aforementioned clinical information, the patient was diagnosed as having acute appendicitis. A CT scan with intravenous contrast was performed to confirm the diagnosis. The scan demonstrated colonic wall thickening with edematous haustral folds suggestive of pseudomembranous colitis. Further, an endoluminal lesion was observed in the cecum with an average size of 6 cm. The lesion was well-defined and had a homogenous fat density with no solid component. The mass was causing a partial colonic obstruction. Such findings conferred the diagnosis of cecal lipoma (Figure 1).

**Figure 1:** Selected axial (A) and coronal (B) CT images of the abdomen demonstrating an endoluminal mass lesion (arrow) in the cecum with homogeneous fat density suggestive of cecal lipoma. Also, note the thickened haustral folds in keeping with pseudomembranous colitis

The patient was prepared for an emergency laparoscopy for further evaluation and management. The operation was done under general anesthesia and the patient was placed in the supine position. Limited segmental rection of the cecum with appendectomy was performed. The estimated blood loss was 10 mL and the total operative time was 100 minutes. The patient tolerated the operation with no complications. He had an uneventful recovery. Histopathological examination of the resected sample revealed the diagnosis of cecal lipoma and the associated acute appendicitis. The patient was discharged on the fifth postoperative day. After 3 months of follow-up, the patient remained asymptomatic with no active issues.

## Discussion

We presented the case of a middle-aged man with acute appendicitis caused by cecal lipoma, a very unusual etiology of acute appendicitis. Colonic lipoma is a rare mesenchymal tumor of the gastrointestinal tract that is composed of well-differentiated adipose tissue. It is reported that colonic lipoma has an incidence of 0.2% [4]. As in the present case, colonic lipoma tends to develop in the right hemicolon, including the cecum and the ascending colon. The pathogenesis of colonic lipoma remains unclear. However, it is suggested that chronic inflammation of the cecum could play a role.

The majority of colonic lipoma cases are asymptomatic and are detected incidentally during colonoscopy or surgery. It is reported that less than 25% of cases of colonic lipoma are symptomatic [5]. The clinical presentations of colonic lipoma include intestinal obstruction, rectal bleeding, and intussusception. In the present case, the presentation of colonic lipoma with acute appendicitis is very rare [6]. The site and size of the lipoma determine the clinical presentation. For instance, lipomas with a size less than 2 cm are usually asymptomatic [7]. It is worth noting that colonic lipoma may pose a diagnostic difficulty and it may be mistaken for malignancy in certain cases [8].

Radiological imaging studies are crucial in making the diagnosis. In the barium fluoroscopic studies, the colonic lipoma appears as submucosal or pedunculated mass with a smooth surface with no ulcers [8]. However, CT and MRI scans can make the diagnosis more readily [9]. In the present case, the CT scan was performed to confirm the diagnosis of acute appendicitis and to rule out any complications like abscess formation. The scan demonstrates a well-circumscribed lesion with complete fat density. The presence of solid components may suggest liposarcoma.

Regarding the management of colonic lipoma, an endoscopic resection is a feasible option for small and pedunculated lesions. However, for tumors larger than 2 cm, surgery is the appropriate management. The type of surgery is determined by the size and site of the lesion [8]. In the present case, local resection of the tumor was performed along with appendectomy during laparoscopy.

## Conclusions

Lipoma is a rare benign tumor of the gastrointestinal tract. Clinicians should maintain a high index of suspicion for benign and malignant neoplasms when they encounter patients with suspected acute appendicitis in the adult population. A CT scan plays a vital role in making the diagnosis and identifying any underlying pathologies. Laparoscopic resection of the colonic tumor is a preferred management approach for large colonic lipomas.
